# Design and Image Research of Tennis Line Examination Based on Machine Vision Analysis

**DOI:** 10.1155/2021/2436120

**Published:** 2021-09-20

**Authors:** Liu Yan, Sun Xin

**Affiliations:** ^1^College of Sports Science, Harbin Normal University, Harbin 150025, China; ^2^Harbin Finance University, Harbin 150030, China

## Abstract

In view of the intelligent demand of tennis line examination, this paper performs a systematic analysis on the intelligent recognition of tennis line examination. Then, a tennis line recognition method based on machine vision is proposed. In this paper, the color region of the image recognition region is divided based on the region growth, and the rough estimation of the court boundary is realized. In order to achieve the effect of camera calibration, a fast camera calibration method which can be used for a variety of court types is proposed. On the basis of camera calibration, a tennis line examination and segmentation system based on machine vision analysis is constructed, and the experimental results are verified by design experiments. The results show that the machine vision analysis-based intelligent segmentation system of tennis line examination has high recognition accuracy and can meet the actual needs of tennis line examination.

## 1. Introduction

Tennis, as one of the hottest ball games, has gained the attention of many fans all over the world. In order to ensure the fairness of tennis match, the third-party evaluators are required to participate in the evaluation of the game, called line review. In the competition, the tennis ball flies very fast, so whether the ball is out of bounds the moment it hits the ground needs scientific evaluation. The traditional line examination is judged by the naked eye, which is controversial. The emergence of “eagle eye” technology further improves the fairness of tennis line examination. At present, eagle eye system is mostly “instant playback” system; that is, in case of dispute, it is judged by applying for playback, and the eagle eye coverage is in advance. Therefore, not all cases can challenge the form of new assessment, so the accuracy and timeliness of current tennis line review need to be further improved [1].

At present, the application of machine vision in sports video analysis is more, mainly in football and basketball. In football and basketball, match support has matured. Although the heat of tennis video analysis is not comparable to football and basketball, its environment is more complex and requires higher quality of machine vision recognition. At present, the requirements of sports video visual recognition are mainly reflected in the above aspects, which are vision, text, and hearing [2]. For tennis, the time detection of tennis video mainly starts from visual information, such as lens type analysis, detection, and tracking of players and court. Tennis competition is affected by the court, angle, and other complex factors, resulting in the judgment result of the ball landing out of bounds. Therefore, high-quality machine vision recognition method is needed for video and image analysis to eliminate complex background interference and improve the accuracy of tennis line review [3].

Based on the above requirement analysis, the image processing technology based on machine vision is proposed. In this paper, combined with the actual needs of tennis line review, the design of tennis line review machine vision assistant system and its effect are analyzed. This article further improves the recognition accuracy of tennis line review through visual and algorithm improvements, which has a certain effect on the development of tennis line review.

## 2. Construction of the Machine Vision Algorithm Model

### 2.1. Model Derivation

It is inevitable that objects with the same color as the court will appear in the video frame of tennis match. Therefore, it is necessary to remove these noncourt factors in the detection of court cashing. In this paper, local entropy is introduced as texture feature, and the uncertainty of random variables is quantitatively processed by entropy. In image processing, entropy can be used to measure image homogeneity, which is expressed as follows [4]:

(1) $$\begin{array}{c} H=-\sum_{i=0}^{255}P_{i}\log\;P_{i},\\ P_{i}=\frac{N_{i}}{N}. \end{array}$$

Here, Ni represents the pixel gray value, N represents the number of pixels with gray value in the region, and Pi represents the probability of gray value of. The main color filtering algorithm is constructed by image local entropy, and its flow can be expressed as the result shown in Figure 1. After filtering the main color, a color filter can be obtained, which is represented as a binary image in the computer. In the image, the pixel with the corresponding value of 1 in the video frame is marked as the main color; otherwise, it is the nondominant color. After that, the local entropy of the video frame can be calculated and processed, the local entropy image binarization processing is carried out through the adaptive threshold, the optimized filter is obtained through the fusion processing, and the main color detection is realized by the filter [5].

On the basis of the above main color filtering algorithm, the frame diagram of the court segmentation system is constructed, as shown in Figure 2. The camera is calibrated by the main color filtering algorithm, and the court sideline is accurately segmented based on the AOC segmentation algorithm [6].

### 2.2. Calibration

The camera calibration process mainly includes three steps: the detection of court sideline, the analysis of court type, and the solution of optimal homography matrix. The model combines with the court sideline detection to obtain the four benchmark points calibrated by the camera. In this paper, the tennis sideline is identified. In the actual recognition, only part of the court area will be identified in real time at a certain time. Therefore, the algorithm complexity can be reduced by reducing the parameter space of the optimal unit matrix solving stage [7]. The tennis court segmentation based on AOC mainly uses the camera calibration results to calculate the proportion of the court part in the court model area and projects the region into the image through the homography matrix and finally obtains the accurate segmentation result. Next, we analyze the algorithm of the process [8].

The working principle of pinhole camera is as follows: light is emitted from a distance and projected into an image plane through the camera pinhole. If the focal length of the camera is *f*, the distance between the camera and the object is *Z*, any point of the object can be expressed as *X*, and the *X* corresponding point on the image plane is *x*; then [9],

(2) $$\begin{array}{c} -{\frac{x}{f}}_{i}=\frac{X}{Z}. \end{array}$$

By exchanging pinholes and image planes, (2) can be expressed as another mathematical expression [10]:

(3) $$\begin{array}{c} {\frac{x}{f}}_{i}=\frac{X}{Z}. \end{array}$$

The reason for the lack of symbol on the left side of equation (3) is that the target image is not inverted after the pinhole is exchanged with the image plane.

In theory, the center point of the image is the main point, which is also the intersection of optical axis and image plane. In fact, the main point is not on the optical axis. By introducing two parameters *c*_*x*_ and *c*_*y*_ and modeling the position offset of the main point relative to the optical axis, the relationship between point *Q*(*X*, *Y*, *Z*) and its projection point (*x*_screen_, *y*_screen_) can be expressed as [11]

(4) $$\begin{array}{c} x_{\text{screen}}=f_{x}\left(\frac{X}{Z}\right)+c_{x},\\ y_{\text{screen}}=f_{y}\left(\frac{Y}{Z}\right)+c_{y}. \end{array}$$

Here, the focal length in horizontal and vertical directions is different because the imaging shape on the pixel meter is rectangular rather than squared.

The process of coordinate transformation can be realized by projection transformation, and the imaging process of camera itself is projection transformation. The point in the real world is transformed into the corresponding coordinates of the camera image through the camera, which can be expressed in mathematical form. It can be realized by a homography matrix. Through DLT (Direct Linear Transform) algorithm, homography matrix can be solved effectively when enough corresponding coordinate points are given. In tennis match, the transformation relation of the sum of the boundary points of the court can be expressed as [12]

(5) $$\begin{array}{c} S\left[\begin{array}{c} u\\ v\\ 1 \end{array}\right]=H\left[\begin{array}{c} x\\ y\\ 1 \end{array}\right]. \end{array}$$

Here, *S* is an invariant nonzero vector ${\left[\begin{array}{ccc} u & v & 1 \end{array}\right]}^{T}$, *x*′ can be expressed as ${\left[\begin{array}{ccc} x & y & 1 \end{array}\right]}^{T}$, $H=\left[\begin{array}{ccc} h_{1} & h_{2} & h_{3}\\ h_{4} & h_{5} & h_{6}\\ h_{7} & h_{8} & h_{9} \end{array}\right]$, and, in this study, *H* is a 3 *∗* 3 matrix. Therefore, if we can find four points (*X*_*i*_ : (*x*_*i*_, *y*_*i*_, 1), *i*=1,2,3,4) in the real court and the corresponding four points (*U*_*i*_ : (*u*_*i*_, *v*_*i*_, 1), *i*=1,2,3,4) in the image, we can solve the homography matrix [13]:

(6) $$\begin{array}{c} \left[\begin{array}{cccccccc} x_{1} & y_{1} & 1 & 0 & 0 & 0 & -x_{1}u_{1} & -y_{1}u_{1}\\ 0 & 0 & 0 & x_{1} & y_{1} & 1 & -x_{1}v_{1} & -y_{1}v_{1}\\ x_{2} & y_{2} & 1 & 0 & 0 & 0 & -x_{2}u_{1} & -y_{2}u_{2}\\ 0 & 0 & 0 & x_{2} & y_{2} & 1 & -x_{2}v_{2} & -y_{2}v_{2}\\ x_{3} & y_{3} & 1 & 0 & 0 & 0 & -x_{3}u_{3} & -y_{3}u_{3}\\ 0 & 0 & 0 & x_{3} & y_{3} & 1 & -x_{3}v_{3} & -y_{3}v_{3}\\ x_{4} & y_{4} & 1 & 0 & 0 & 0 & -x_{4}u_{3} & -y_{4}u_{4}\\ 0 & 0 & 0 & x_{4} & y_{4} & 1 & -x_{4}v_{3} & -y_{4}v_{3} \end{array}\right]\left[\begin{array}{c} h_{1}\\ h_{2}\\ h_{3}\\ h_{4}\\ h_{5}\\ h_{6}\\ h_{7}\\ h_{8} \end{array}\right]=\left[\begin{array}{c} u_{1}\\ v_{1}\\ u_{2}\\ v_{2}\\ u_{3}\\ v_{3}\\ u_{4}\\ v_{4} \end{array}\right]. \end{array}$$

Thus, the homography matrix can be obtained.

In the process of storing the golf course model, it is necessary to store the position of the court boundary line, which is usually realized by the way of configuration file storage. In this paper, the configuration file is stored in the format of key value, which mainly includes three attributes, namely, tennis court height (field), tennis court width (field), and the tennis field. According to the position of the sideline, it can be divided into left court boundary (field lines) and right field. With this setting, it is easy to search some frames in a centralized way. On this basis, the court can be further divided into horizontal lines and vertical lines. The boundaries of each line are shown in the model standard format: line = “(*x*_1_*Y*_1_), (*x*_2_*Y*_2_)” [14].

In the calibration process, four lines (horizontal line and vertical line are both two) are selected from the field model for calibration. In order to avoid repeated calculation of calibration points, the vertical line should be sorted from left to right, and the horizontal line from top to bottom. For the straight line of the court model, you can control the field in the configuration file. The lines set is sorted by manually planning the line order. It can be sorted only once, while the straight lines in the image can be sorted according to the distance between these lines and the datum point, which is represented as *ω*. Set the reference point as the midpoint of the left boundary and the key point of the upper boundary of the image, as shown in Figure 3 [15].

The horizontal line of the image is represented as *h*_1_, and the vertical line of the image is represented as *v*_1_. The horizontal and vertical lines in the model are represented as *h*_1_′ and *h*_2_′, respectively. The subscript of the line is set according to the distance from the line to the reference point. If the central line of the set of horizontal lines exists, *ω*(*h*_*l*_) ≥ *ω*(*h*_*l*+1_), as shown in Figure 4 [16].

When solving the optimal homography matrix, it is mainly realized by processing all line combinations. Specifically, two horizontal lines are randomly obtained from the image set, which are represented as *h*_*i*_ and *h*_*k*_, respectively, and the two horizontal lines are randomly returned from the established tennis court model and are, respectively, represented as *h*_*i*_′ and *h*_*k*_′, *i* > *k*. The same method is used to obtain two points from the tennis court image and the tennis court model, and a combined image is obtained through the intersection of two and two, and the four intersection points are calculated, as shown in the following formula [17]:

(7) $$\begin{array}{c} p_{1}=h_{i}\times v_{m},\\ p_{2}=h_{i}\times v_{n},\\ p_{3}=h_{k}\times v_{m},\\ p_{4}=h_{k}\times v_{n}. \end{array}$$

The image is subdivided into the left and right court modes for space reduction, but the overall parameter size is still large; if the algorithm detects more than one straight line, this will lead to a rapid increase in data volume, resulting in a longer data calculation time, and finding the results of model parameters is more time-consuming;, the actual application of the algorithm is not good and obviously cannot meet the timely needs of tennis tournaments; in order to improve the efficiency of tennis line review, further improvement is needed [18].

When there are many parameters in the model, it is difficult to find the optimal solution. Therefore, this paper uses the method of not seeking *H* matrix and other follow-up operations to improve the efficiency of solving the optimal solution. Two pruning methods are introduced in the system to reduce the time complexity and eliminate the obvious errors in the system calculation process.

The first method of pruning is to estimate the height of the court through two image horizontal lines and the corresponding horizontal lines in the corresponding model. If the actual heights of the two images are too far, they will be discarded directly, and the vertical lines will be operated the same way. Through this pruning method, the score calculation of homography matrix solution can be effectively avoided, and the amount of calculation can be reduced [19].

Another pruning method is to get the homography matrix by calculating the calibration set of the system. The homography matrix itself is estimated. It is obviously impossible to obtain the value of the optimal solution by discarding the homography matrix. Although this process is accompanied by the calculation of the homography matrix, the calculation process is fast. In the process of image processing, it is necessary to reflect the golf course model to the corresponding image of the model. The mapping process is one-to-one corresponding, so there is a certain time loss in the process.

There are eight degrees of freedom in the homography matrix, which are camera internal parameter ^*∗*^ 3, camera rotation ^*∗*^ 3, translation parameter ^*∗*^ 1, and focal length parameter ^*∗*^ 1. The remaining parameters are related to different directional scaling; that is, the horizontal and vertical directions show different zoom ratios in the process of zooming. The camera imaging process can be expressed as [20]

(8) $$\begin{array}{c} p_{i}=Hp_{i}^{\prime }=\left[\begin{array}{ccc} f & 0 & o_{x}\\ 0 & f & o_{y}\\ 0 & 0 & 1 \end{array}\right]\left[\begin{array}{cccc} r_{00} & r_{01} & r_{02} & t_{x}\\ r_{10} & r_{11} & r_{12} & t_{y}\\ r_{20} & r_{21} & r_{22} & t_{z} \end{array}\right]\left[\begin{array}{cccc} 1 & 0 & 0 & 0\\ 0 & \beta & 0 & 0\\ 0 & 0 & 1 & 0\\ 0 & 0 & 0 & 1 \end{array}\right]\left[\begin{array}{c} x^{\prime }\\ y^{\prime }\\ z^{\prime }=0\\ 1 \end{array}\right]. \end{array}$$

Here, the focal length is denoted by *f*. In fact, the anisotropic scaling can be ignored in the real world, so *β* can be set to 1, which is one of the basic conditions for pruning.

### 2.3. The Tennis Court Is Precisely Divided

In this paper, the model is designed to accurately divide the side of the court for the needs of tennis wire review, and the process divides the court by a single matrix, which mainly consists of two parts, namely, AOC calculation and AOC reverse projection. AOC is defined as the area captured by the camera. In tennis, the camera is not filmed in the whole process. In order to improve the identification effect of the court, the local area is generally shot in high definition to improve the effect of line inspection. Therefore, by calculating AOC, the precise division of the pitch boundary can be achieved. AOC's calculation process consists of four main steps, namely, coordinate mapping, field shape boundary recognition, coordinate detection, and AOC generation. Mapping coordinates to a model image results in a standard shape pitch boundary model after projection, due to different camera angles, or produces two types of polygon shapes, as shown in Figure 5 [21].

The projection point under the top view angle is represented as (*P*_*i*1_′, *P*_*i*2_′, *P*_*i*3_′, *P*_*i*4_′), and the top point of the court under the top view angle is represented as (*P*_*T*1_, *P*_*T*2_, *P*_*T*3_, *P*_*T*4_). (*P*_*i*1_′, *P*_*i*2_′, *P*_*i*3_′, *P*_*i*4_′), the connecting lines of the vertices, form a convex polygon or a self-intersecting polygon. The two situations are identified, respectively. If the result is a convex polygon, *A*_*i*_ is used to represent the coincidence area between the polygon and the court; otherwise, *A*_*i*_ is used to represent the coincidence area between the polygon extension line and the court.

In order to solve problem *A*_*i*_, we need to calculate three point sets. First, we calculate the projection to get the polygon (*P*_*i*1_′, *P*_*i*2_′, *P*_*i*3_′, *P*_*i*4_′) and the intersection point of the court boundary. Second, the tennis court vertex (*P*_*i*1_′, *P*_*i*2_′, *P*_*i*3_′, *P*_*i*4_′) in the polygon area is searched, and then the four vertices in the tennis court are searched. The rearrangement of these points is completed by AOC generation process. Every two adjacent vertices form an edge of the polygon. In both cases, the point set can be represented as (*Q*_*i*_, *P*_*i*2_′, *P*_*i*3_′, *P*_*i*4_′, *P*_*T*3_) and (*Q*_*i*_, *P*_*i*2_′, *P*_*i*3_′, *P*_*i*4_′, *Q*_2_), respectively.

AOC reverse projection is carried out after rearing, which is the last step in the operation of the model, and the single matrix results are projected back to the model image, resulting in a more accurate reverse projection result, thus obtaining the field boundary distribution result.

## 3. Image Processing

Although the image is grayed, filtered, and threshold-segmented, there are still some small particles in the image and the contour is not clear. Therefore, it is necessary to process the image morphology. Image morphology mainly removes the unwanted information from binary image and strengthens the needed information. Morphological processing is mainly divided into pixel morphological processing and regional morphological processing. It can be seen from the image after threshold segmentation that there are pixels in the contour of the target which should be the target but divided into background points. At the same time, there are pixels that should be background but are divided into targets. Therefore, morphological processing should be carried out on these misjudged pixels first. The morphology of image is similar to image filter operator. It is to replace the original pixel with a certain shape of structural elements and pixels in the domain and then study the feature information of the image. The basic treatment of morphological treatment is corrosion and expansion, and another form of morphological processing is based on corrosion and expansion.

### 3.1. Corrosion

Corrosion is to move the corrosion element from left to top and from top to bottom in image A. Only when it is the same as the structure element will it be retained, and different places will be removed. The etching of binary image with structural element B can be expressed as follows.

*B*(*x*) is the structural element and A is the original image. The corrosion of gray scale image can be expressed by the following formula:

(9) $$\begin{array}{c} A\Theta B=\left\{x|B\left(x\right)\subseteq A\right\},\\ \left(f\Theta b\right)=\min\left\{f\left(s+x,t+y\right)-b\left(x,y\right)|\left(s-x,t-y\right)\notin D_{f};\left(x,y\right)\in D_{b}\right\}. \end{array}$$

Corrosion is mainly used to eliminate the high brightness of the isolated pixels in the image, which can refine the contour of the target. As a result, the high brightness area of the image becomes smaller and the dark brightness area is expanded.

### 3.2. Expansion

In contrast to dilation and erosion, when traversing all pixels in image A, as long as the intersection with structural elements is not empty set, the binary image expansion can be expressed by the following formula:

(10) $$\begin{array}{c} \left(f\Theta b\right)=\max\left\{f\left(s-x,t-y\right)+b\left(x,y\right)|\left(s-x,t-y\right)\notin D_{f};\left(x,y\right)\in D_{b}\right\}. \end{array}$$

Dilation can fill the holes and gaps of the image and also can expand the outline of the image. For the gray image, it can expand the brightness area and shrink the dark brightness area.

### 3.3. Hole Filling

Hole filling is an algorithm based on set expansion, complement, and intersection. The main process of hole filling is to seed a background pixel in the image boundary. According to the principle of 8-connected, foreground 1 is used to fill the background outside the particle, and then the image filled with background is reversed to obtain the hole image represented by foreground color *L*. The hole filling can be completed by adding the hole image represented by foreground color *L* and the original binary image. It can be expressed as follows:

(11) $$\begin{array}{c} X_{k}=\left(X_{k-1}⊕B\right)\cap A^{c}\\ k=1,2,3,\cdots . \end{array}$$

### 3.4. Morphological Treatment of Granules

Particles refer to the region composed of nonzero or high gray pixels connected with each other in the image. Particle morphology processing includes particle separation, image labeling, particle region division, and particle filtering. In this paper, the image is filtered by two values, that is, the particle size and the particle area. Users can choose the filtering standard according to different needs. In this paper, the nontarget particles in the image are removed according to the particle area.

The edge of an image refers to the pixels with mutation in the image, which can be connected to form the outline of the image. Edge detection can be completed by one or two derivatives. The main detection algorithms are gradient detection, Robert detection, Sobel detection, Prewitt detection, and canny detection.

#### 3.4.1. Gradient Detection

Gradient operator is calculated by calculating partial derivatives ∂*f*/∂*x* and ∂*f*/∂*y* of each pixel in the image. For partial derivatives, it can be approximately expressed as

(12) $$\begin{array}{c} \frac{\partial f}{\partial x}=f\left(x+1\right)-f\left(x\right),\\ \frac{\partial f}{\partial y}=f\left(y+1\right)-f\left(y\right). \end{array}$$

Then, the gradient operator can be expressed as follows:

(13) $$\begin{array}{c} g_{x}=\frac{\partial f\left(x,y\right)}{\partial x}=f\left(x+1,y\right)-f\left(x,y\right),\\ g_{y}=\frac{\partial f\left(x,y\right)}{\partial y}=f\left(x,y+1\right)-f\left(x,y\right). \end{array}$$

#### 3.4.2. Roberts Operator

Robert crossover operator can extract the edge in diagonal direction. Suppose that there is a region of size 3 × 3, in which the element is *a*_*ij*_, and the operator can be expressed as follows:

(14) $$\begin{array}{c} g_{x}=\frac{\partial f}{\partial x}=\left(a_{33}-a_{22}\right),\\ g_{y}=\frac{\partial f}{\partial y}=\left(a_{32}-a_{23}\right). \end{array}$$

Robert operator is used to extract the image contour. Compared with the gradient operator, the edge is well extracted, and the contour extraction is continuous. Although it looks a little discontinuous from the diagram, it is a continuous boundary after zooming in.

#### 3.4.3. Prewitt Operator

Prewitt operator is improved from Robert operator. Prewitt operator takes into account the property of center point to end data and has more information about edge direction. For a region of 3 × 3 size, the element is *a*_*ij*_. The Prewitt operator can be used to represent the following:

(15) $$\begin{array}{c} g_{x}=\frac{\partial f}{\partial x}=\left(a_{31}+2a_{32}+a_{33}\right)-\left(a_{11}+2a_{12}+a_{13}\right),\\ g_{y}=\frac{\partial f}{\partial y}=\left(a_{13}+2a_{23}+a_{33}\right)-\left(a_{11}+2a_{21}+a_{31}\right). \end{array}$$

### 3.5. Canny Operator

Canny operator is the most excellent operator among the basic edge detectors. Firstly, Canny operator smoothes the image with a Gaussian filter. Let *G*(*x*, *y*) represent the Gaussian function and represent input images; then smoothing the input image can be expressed as

(16) $$\begin{array}{c} g\left(x,y\right)=G\left(x,y\right)\cdot f\left(x,y\right),\\ G\left(x,y\right)=e^{-\left(x^{2}+y^{2}/2\sigma^{2}\right)}. \end{array}$$

The second step is to calculate the gradient value and angle of the image:

(17) $$\begin{array}{c} M\left(x,y\right)=\sqrt{{\left(\frac{\partial g\left(x,y\right)}{\partial x}\right)}^{2}+{\left(\frac{\partial g\left(x,y\right)}{\partial y}\right)}^{2}},\\ \alpha \left(x,y\right)=\arctan\left[\frac{\partial g\left(x,y\right)/\partial x}{\partial g\left(x,y\right)/\partial y}\right]. \end{array}$$

The third step is to carry out nonmaximum suppression on the gradient amplitude image and compare the horizontal angle of −45° and vertical angle of +45° with the image to find the closest angle direction. If the amplitude is at least less than one of the two neighbors of the closest angle direction, then *g*_*N*_(*x*, *y*)=0 (suppression), and then *g*_*N*_(*x*, *y*)=*M*(*x*, *y*), so as to obtain the image after nonmaximum suppression, that is, *g*_*N*_(*x*, *y*).

The last step is to use double threshold processing and connection analysis to detect and connect edges. The processing of low threshold *T*_*L*_ and high threshold *T*_*H*_ can be regarded as the addition of two images as follows:

(18) $$\begin{array}{c} g_{NH}\left(x,y\right)=g_{N}\left(x,y\right)\geq T_{H},\\ g_{NH}\left(x,y\right)=g_{N}\left(x,y\right)\geq T_{H}. \end{array}$$

At the beginning, the pixel values of the two images are set to zero. After threshold processing, the nonzero pixels in the high threshold image are removed by subtracting the low threshold image from the high threshold image, and the strong pixels in the high threshold image will be marked as edge pixels.

In Canny operator, we can change the value of *O*, low threshold, high threshold, and window size to achieve the purpose of contour extraction. Canny operator can extract contour well, but it takes more time.

### 3.6. The Contour Is Extracted by Morphological Processing

Morphological contour extraction is based on the evolution of corrosion expansion, and there are two main extraction methods: inner gradient boundary and outer gradient boundary. If *A* is used to represent the original image, *B* is the structural element, and *β*(*A*) is the boundary of image A, and then the inner and outer gradient boundaries can be expressed as follows:

(19) $$\begin{array}{c} \beta \left(A\right)=A-\left(A\Theta B\right),\\ \beta \left(A\right)=\left(A⊕B\right)-A. \end{array}$$

It can be seen from the formula that the inner gradient boundary first etched image *A* with structural element *B*, and then the boundary can be obtained by subtracting the corroded image with image *A*. The extraction of external gradient is to expand image *A* with structuring element *B* first and then subtract image *A* from the expanded image to obtain the outer gradient boundary. Different choices of structural elements can achieve different effects. The larger the structure element is, the thicker the boundary will be.

Compared with these six methods, the gradient operator, Sobel operator, and Prewitt operator can extract the contour, but the contour is not continuous, and further processing is needed. Roberts operator, Canny operator, and morphological extraction can extract the contour of the target completely. Although Canny operator is the best operator, it consumes more time and increases the processing time of machine vision system. Roberts operator can also extract the contour, but the contour extraction has a little dilation effect, which will cause errors for the next measurement; and morphology can well propose the contour of the target, so this paper selects the contour extraction of morphology.

## 4. Model Construction

Based on the detection and image processing of the front-end tennis court, the requirements of the line review of the tennis court are analyzed and the system prototype is designed. The system constructed in this paper mainly designs a structure with three tiers, which are application layer, data access layer, and data connection layer. The hierarchical structure of the overall design of the system is shown in Figure 6:

1. The application layer is the application process of sports video moving object detection and tracking system. It is mainly the data used when users access sports video management module, video acquisition management module, target detection management module, and target tracking management module.
2. The data access layer is the process of accessing data in the system. The sports video moving object detection and tracking system uses the target tracking and target detection algorithm to access the data in the database.
3. The data connection layer is used to store the data information in the system, such as video information, user information, video detection information, and video tracking information. The functional structure of the system is shown in Figure 7.

The target detection management function is to detect and analyze the target in the sports video collected, which can be used as the analysis data in the training. The main executors of this function are video analysis users. This function mainly includes four functions: target detection, target model establishment, target model updating, and detection result display. The target detection diagram is shown in Figure 8. Firstly, the video analysis manager enters the video target detection management module with his username and password and then submits the video target detection request. After the detection is completed, the detection results are displayed.

## 5. Experimental Analysis

In order to verify the validity of the model, this paper collects the video design experiment of tennis match from the Internet, selects multiple sets of image frames from the video as the test set, and compares the algorithm with the histogram method and the hybrid Gauss model. These image frames are recognized by the test set images to compare the final recognition results. Firstly, the extraction effect of primary colors was analyzed. The accuracy test results of different primary colors were shown in Table 1 and Figure 9. It can be found from the test results that the model built in this paper has a remarkable effect; the analysis is that the system in this paper will constantly update the parameters in its operating sheet and filter out some color interference.

Next, divide the field of the model area to determine whether the tennis ball falls outside the divided limit area. Taking each selected video frame as the test set, the court and the main color region recognition method are studied through the AOC method. When the tennis ball is determined, since all the hitting results in the video frame are known, the recognition results can be compared with the actual results in order to get the recognition accuracy.

After expanding the experiment, the identification of whether the tennis ball's landing moment was out of boundary was judged on the basis of the AOC method and the main color area method, respectively, and the results are shown in Table 2 and Figure 10.

From the above graph segmentation results, the recognition method based on the main color region belongs to a rough recognition algorithm. For tennis competition, the environment of the court is more complex, so it is difficult to get more accurate recognition results only through this method. The recognition algorithm based on AOC is more accurate, and the identification results can be effectively improved by calibrating the camera to meet the actual needs of tennis line review.

## 6. Conclusion

This paper analyzes the accuracy of traditional tennis line review and proposes an intelligent recognition model of tennis line review based on AOC with the support of machine vision algorithm and verifies the performance of the model. The process of coordinate transformation can be realized by projection transformation, and the imaging process of camera itself is projection transformation. The point in the real world is transformed into the corresponding coordinates of the camera image by the camera. The process can be expressed in mathematical form and realized by a homography matrix. The model designed in this paper can accurately segment the sideline of tennis court according to the needs of tennis line review. The process divides the course by homography matrix, which includes two parts: AOC calculation and AOC back projection. The performance analysis of the model constructed in this paper shows that the recognition algorithm based on AOC is more accurate. By calibrating the camera, the recognition results can be effectively improved to meet the actual needs of tennis line review.

This paper only conducts system performance verification through theoretical research and a small number of image experiments, so it is necessary to further expand the research and practice, and, in the follow-up research, it is necessary to verify the system in combination with actual competitions.

## Figures and Tables

**Figure 1:** Main color filtering algorithm flow.

**Figure 2:** Stadium segmentation system.

**Figure 3:** The tennis court line is sorted.

**Figure 4:** Acquisition of a fixed point.

**Figure 5:** Two types of AOC.

**Figure 6:** Hierarchical structure of the overall system design.

**Figure 7:** Overall function structure of the system.

**Figure 8:** Collaboration diagram of target detection function.

**Figure 9:** Comparison of the accuracy of the main color extraction.

**Figure 10:** Comparison of the accuracy of the identification method.

**Table 1:** Comparison table of the accuracy of the main color extraction.

Video sequence group	Histogram method (%)	GMM method (%)	Method of this article (%)
1	81.51	85.29	91.42
2	94.67	94.51	97.97
3	87.20	89.04	95.69
4	93.15	95.60	98.73
5	86.38	88.42	89.95

**Table 2:** A comparison table of the accuracy of the identification method.

The video sequence	A field boundary detection algorithm based on the main color area (%)	AOC-based pitch segmentation algorithm (%)
Tennis video 1	84.21	97.44
Tennis video 2	92.42	98.34
Tennis video 3	89.53	98.76
Tennis video 4	88.43	97.65
Tennis video 5	89.51	98.35

## Data Availability

The data used to support the findings of this study are available from the corresponding author upon request.
